# A Study on Curcumol Influencing Proliferation and Apoptosis of Hepatocellular Carcinoma Cells through DJ-1/PTEN/PI3K/AKT Pathway

This article has been retracted.

**DOI:** 10.1155/2022/9912776

**Published:** 2022-05-20

**Authors:** Rongzhen Zhang, Lu Zhong, Kewei Sun, Jiao Liu, Qianna Wang, Dewen Mao, Gang Fang, Fuli Long

**Affiliations:** ^1^Graduate School of Hunan University of Chinese Medicine, Hunan 410208, China; ^2^Hepatology Department, First Affiliated Hospital, Guangxi University of Chinese Medicine, Guangxi 530023, China; ^3^Ruikang Clinical Faculty, Guangxi University of Chinese Medicine, Guangxi 530011, China; ^4^Hepatology Department, First Affiliated Hospital, Hunan University of Chinese Medicine, Hunan 10202, China; ^5^Graduate School, Guangxi University of Chinese Medicine, Guangxi 530001, China; ^6^Zhuang Medicine College, Guangxi University of Chinese Medicine, Guangxi 530001, China

## Abstract

**Objective:**

To study the mechanism of curcumol affecting the proliferation and apoptosis of liver cancer cells through the DJ-1/PTEN/PI3K/AKT pathway.

**Method:**

HepG2 cells were cultured in vitro, treated with curcumol at concentrations of 10, 30, and 100 *μ*g/mL, and DMSO was used as a control. The levels of cell proliferation and apoptosis were measured by CCK-8 and flow cytometry, respectively. RT-PCR and western blot were used to detect PTEN, p-AKT, DJ-1, and PI3K gene and protein expression changes.

**Result:**

(1) Compared with the DMSO blank control group, the proliferation level of liver cancer cells in the 10 *μ*g/mL curcumol group decreased, and the proportion of apoptosis increased (p <0.05). (2) Compared with the blank control group and the 10 and 30 *μ*g/mL concentration groups, the proliferation level of liver cancer cells in the 100 *μ*g/mL curcumol group was significantly reduced, and the proportion of cell apoptosis was significantly increased (*p* < 0.05). (3) Curcumol can significantly increase the expression of PTEN gene and protein in liver cancer cells and reduce the expression of DJ-1 and PI3K genes and protein in liver cancer cells (*p* < 0.05).

**Conclusion:**

Curcumol can regulate DJ-1, PTEN, PI3K, and AKT signal transduction pathways, inhibit cell proliferation, and cause a significant increase in the proportion of cell apoptosis, and the pharmacodynamic effect of curcumol is dependent on the time and dose of action.

## 1. Introduction

The occurrence of hepatocellular carcinoma is a complex multistage process in which gene mutation may be triggered when normal tissue cells are subjected to injury, external induction, or microenvironment change, causing oncogene activation, antioncogene inactivation, etc., thereby leading to the generation of cancer cells in the body. The cancer cells can gradually proliferate at the site of origin to grow into primary tumor, or partial cancer cells migrate toward surrounding or distant tissues after leaving the primary tumor, thus forming metastatic tumors [1–5]. In addition, hepatocarcinogenesis and development are the processes of cell hyperproliferation and inhibited apoptosis of cells, which complement proliferation and collectively maintain the stability of cell numbers in organ tissues. Normal liver cancer epithelial cells exist in programmed death to clear senescent cells, maintaining mucosal cell physiological balance. When various factors cause excessive accumulation of epithelial cells in liver cancer, they have the potential to cause carcinogenesis. Therefore, regulating the proliferation/apoptosis ratio of HCC cells is of great significance for the clinical treatment of HCC [6, 7].

As an active component extracted from traditional Chinese medicine zedoary, curcumol exerts anti-inflammatory and antitumor effects in the body through many mechanisms. Some studies have manifested that curcumol is capable of killing or inhibiting tumor cells in multiple ways, of which the possible mechanism of action involves the induction of cell apoptosis by regulating signaling pathways. However, the specific mechanism of action has not been clarified yet [8].

Recently, research evidence has revealed that DJ-1 plays a certain role in the occurrence of human tumors. It is a type of protein containing 189 amino acids, which was initially identified as an oncogene binding to Harvey-rat sarcoma (H-Ras) and can transform mouse NIH3T3 cells [9]. DJ-1 protein has been found in a variety of malignant tumor cells, including prostate cancer, non-small-cell lung cancer, laryngeal cancer, ovarian cancer, and cervical cancer, and it plays a vital role in promoting cell proliferation and metastasis [10–13]. Several studies have indicated that DJ-1 protein expression is reduced after the human lung cancer NCI-H157 cell line is treated with paclitaxel and MEK inhibitor U0126. The above results illustrate that DJ-1 protein has crucial physiological functions in multiple tumors. However, the role of DJ-1 in the occurrence and development of hepatocellular carcinoma has not been investigated so far.

In this research, curcumol was applied to treat the hepatocellular carcinoma cells, and its inhibitory effect on the proliferation of those cells was examined, so as to further explore its mechanism of action.

## 2. Materials and Methods

### 2.1. Cell Culture and Treatment

Human hepatocellular carcinoma HepG2 cell lines in the logarithmic phase were fetched and digested with 0.25% trypsin, which were then inoculated into a cell culture plate. The cells in the experimental group were treated with different concentrations of curcumol, and those in the control group were added with dimethyl sulfoxide (DMSO) in the same volume. After that, all the cells were cultured for 24, 48, and 72 h, respectively, for subsequent experiments and studies.

### 2.2. Western Blotting

The HepG2 cells cultured for different time periods were fetched and lysed to extract the total protein. After the protein concentration was measured using BCA method, the appropriate protein concentration was explored, followed by loading, electrophoretic separation of protein, membrane transfer via Bio-Rad system, and sealing in skim milk powder. Next, DJ-1, phosphatase and tensin homolog deleted on chromosome ten (PTEN), phosphorylated p-Akt, phosphatidylinositol 3-kinase (PI3K), and *β*-actin antibodies were added for incubation overnight; then, the membrane was washed, secondary antibodies were added for color development, and the ECL system was utilized to record the results.

### 2.3. Quantitative Real-Time Polymerase Chain Reaction (RT-PCR)

Quantitative RT-PCR was performed to detect the gene expression level of the HepG2 cells. The HepG2 cells treated with varying concentrations of curcumol for different time periods were taken to extract the total ribonucleic acid (RNA), and cDNA was obtained using a reverse transcription kit for amplification test. Next, nontemplate control and positive control were set up for quality control, quantitative RT-PCR was conducted in triplicate with *β*-actin as the loading control, and the 2^-*ΔΔ*Ct^ method was adopted to calculate and analyze all the expressions (Table 1).

### 2.4. Detection of Cell Proliferation Inhibition via Cell Counting Kit-8 (CCK-8) Assay

The cultured cells were prepared into single-cell suspension after digestion with trypsin, counted, and inoculated into a 96-well cell culture plate with 100 *μ*L 5 × 10^3^ cells in each well according to the operation manual. Next, CCK-8 was applied to measure the impacts of curcumol in varying concentrations and different treatment times on the proliferation activity of the HepG2 cells. The cell culture plate was taken out at regular intervals to determine the absorbance at the wavelength of 450 nm using a microplate reader, of which the DMSO treatment group was regarded as the control. Proliferation inhibition rate (%) = [1 − optical density (OD)_experimental group_/OD_DMSO_] × 100%.

### 2.5. Detection of Cell Apoptosis via Flow Cytometry

The flow cytometry was performed to detect the cell apoptosis, and the apoptotic cells and living or necrotic cells were determined by virtue of Annexin V-fluorescein isothiocyanate (FITC) and propidium iodide (PI). 10 *μ*L Annexin V-FITC and PI staining solution were added separately and incubated in ice bath away from the light for at least 0.5 h, and then, labeled samples were washed twice with precooled phosphate-buffered saline (PBS), and the cell concentration was adjusted to 10^6^/200 *μ*L. The flow cytometer was adopted for analysis.

### 2.6. Data Statistics and Analysis

Statistical Product and Service Solutions (SPSS) 17.0 software was used for all the data, and Student's *t*-test was performed for statistical analysis. *p* < 0.05 suggested that the difference was statistically significant.

## 3. Results

### 3.1. Effects of Curcumol in Varying Concentrations and Different Treatment Times on the Apoptosis of Human Hepatocellular Carcinoma HepG2 Cells

According to the cell apoptosis test, curcumol was able to regulate the physiological functions of the cells and induce cell apoptosis in comparison with the control group (Figure 1 and Table 2). The percentage of early apoptotic cells and late apoptotic cells was 4.39 ± 0.67% and 6.14 ± 1.76% in the 100 *μ*g/mL group treated for 24 h and 1.54 ± 0.52% and 1.31 ± 0.33% in the 10 *μ*g/mL group treated for 24 h, respectively, with significant differences between the two groups (*p* < 0.05), suggesting that the percentage of apoptotic cells is prominently correlated with the drug concentration. In addition, the percentage of early apoptotic cells and late apoptotic cells was 9.27 ± 1.64% and 11.35 ± 2.09%, respectively, in the 100 *μ*g/mL group treated for 72 h, and that was 4.35 ± 0.63% and 5.24 ± 0.86%, respectively, in the 10 *μ*g/mL group treated for 72 h. These results imply that the apoptotic level of hepatocellular carcinoma cells is elevated markedly with the prolongation of treatment with curcumol.

### 3.2. Inhibition of Curcumol in Varying Concentrations and Different Treatment Times on the Growth of Human Hepatocellular Carcinoma HepG2 Cells

The results of HepG2 cell proliferation detected via CCK-8 showed that the cell growth and proliferative capacity were suppressed in the 10*μ*g/mL group, of which the inhibition rate of cell growth and proliferation was 5.25 ± 0.64% at 24 h and 13.35 ± 2.14% at 72 h (Table 3). The inhibitory effect on the cell growth and proliferative capacity was the strongest in the 100*μ*g/mL group, with inhibition rates of 12.36 ± 2.35% and 31.45 ± 3.97% at 24 h and 72 h, respectively. There were significant differences among groups treated with different concentrations of curcumol at the same time point (*p* < 0.05). Moreover, there were also significant differences at different treatment time points in the group treated with the same concentration of curcumol (*p* < 0.05). The above results suggest that the inhibitory effect of curcumol on the growth of human hepatocellular carcinoma HepG2 cells is influenced by its concentration and treatment time.

### 3.3. Effects of Curcumol in Varying Concentrations and Different Treatment Times on Related Protein Expressions to Human Hepatocellular Carcinoma HepG2 Cells

According to western blotting results, DJ-1 protein expression was downregulated in the group treated with 10 *μ*g/mL curcumol compared with the DMSO group (Figure 2, Table 4). With the extension of treatment time, the activity of p-Akt declined continuously, the expression level of PI3K kept decreasing, and the expression level of PTEN rose constantly, displaying significant differences (*p* < 0.05). The effect of downregulating DJ-1 protein expression was more prominent in the group treated with 100 *μ*g/mL curcumol, and as the time was prolonged, p-Akt expression level was reduced constantly, with significant differences among different groups (*p* < 0.05).

### 3.4. Effects of Curcumol in Different Concentrations and Different Treatment Times on Gene Expressions in Human Hepatocellular Carcinoma HepG2 Cells

RT-PCR results manifested that compared with those in the DMSO group, the messenger RNA (mRNA) expression level of PTEN gene was elevated in the group treated with 10*μ*g/mL curcumol. The expression level of DJ-1 gene declined continuously, and that of PTEN gene rose constantly along with the increased treatment time, displaying significant differences (*p* < 0.05). In the 100 *μ*g/mL group, there were significant differences in the changes in mRNA content of PI3K, PTEN, and DJ-1 genes (*p* < 0.05). However, the change in mRNA content of Akt gene was not remarkable (*p* > 0.05) (Table 5).

## 4. Discussion

In this research, the pharmacodynamic and antitumor effects of curcumol, as well as its possible mechanism of action, were investigated, so as to provide information for search of novel anticancer drugs and action targets from traditional Chinese medicine. Curcumol was applied to treat the hepatocellular carcinoma cells to explore whether it could control the expression of DJ-1 and further alter the PI3K pathway through regulating the function of tumor suppressor gene PTEN, thereby exerting the effects of inhibiting tumor proliferation.

Some studies have argued that DJ-1 mediates cell proliferation by upregulating protein kinase B (PKB)/Akt, thus becoming conducive to tumorigenesis [14]. DJ-1 was initially cloned from the protooncogene of NIH-3T3 cells, which is capable of binding to and interacting with H-Ras to perform the regulatory functions of RNA-protein interaction. It can also be isolated from autosome-related genes of early-onset Parkinson's disease (PD). Several categories of DJ-1 site mutation have been discovered in PD patients so far, including the mutation in the C-terminus spirochaete of DJ-1 with deletion of the first five exons (L166P) and mutation of exon 1, intron 4, and exon 5. A number of studies have manifested that DJ-1 also plays a very important role in the occurrence of human tumors. It is reported that the levels of DJ-1 and DJ-1 autoantibody are increased evidently in patients with breast cancer compared with those in healthy population. The content of DJ-1 protein is found to be elevated markedly in primary non-small-cell lung cancer. In spite of large quantities of studies on DJ-1, however, its physiological action still remains unclear to a great extent.

According to CCK-8 assay in this research, curcumol could effectively attenuate the growth of human hepatocellular carcinoma HepG2 cells. It was revealed that as for the hepatocellular carcinoma HepG2 cells treated with different doses of curcumol, the inhibitory effects on cell proliferation became more prominent with the extension of time. Moreover, the pharmacodynamic effect of curcumol was directly proportional to time, and it was also correlated with dose. In addition, it was found in this research that the apoptosis of the HepG2 cells was increased remarkably after curcumol treatment, indicating that curcumol may not only repress cell proliferation but also induce cell apoptosis to a certain extent.

In order to further clarify the potential antitumor mechanism of curcumol, the signaling pathways possibly involved were investigated. PTEN (MMAC/TEP1) is one of the most common mutant-type tumor suppressor genes of human cancers [15], and the PI3K signaling pathway, PKB/Akt signaling pathway, and PTEN signaling pathway are fairly conservative in the whole evolutionary process. Some studies have demonstrated that the upregulation of DJ-1 expression level can antagonize the tumor suppressor gene PTEN, suppress its activity, and ultimately promote the proliferation of tumor cells. In this research, the results of western blotting and RT-PCR indicated that curcumol treatment could trigger the downregulation of DJ-1 protein and gene expressions and constantly increase the content of PTEN protein and gene. PTEN is an essential negative regulator in the PI3K signaling pathway [16, 17]. Furthermore, the inhibited PTEN function can lead to disorders of the PI3K/Akt signaling pathway and overactivation of the signal transduction pathways [18, 19]. p-Akt exerts vital effects in many signal transduction pathways such as cell proliferation, apoptosis, and transcription [20].

According to this research, curcumol was able to act on the DJ-1/PETN/PI3K/Akt signaling pathway and repress Akt activation, thus accelerating cell apoptosis. In addition, such functions had significantly time- and dose-dependent effects. In other words, the antitumor effect of curcumol was enhanced markedly along with increases in time and dose. The abovementioned results suggest that curcumol can exert a certain antitumor effect, which may be a candidate antitumor drug.

## Figures and Tables

**Figure 1:** Effects of curcumol on percentage of apoptotic human hepatocellular carcinoma HepG2 cells at 24 h after administration: (a) control group, (b) 100 *μ*g/mL group, (c) 30 *μ*g/mL group, and (d) 10 *μ*g/mL group.

**Figure 2:** Effects of curcumol in varying concentrations on protein expressions in human hepatocellular carcinoma HepG2 cells at 24 h after administration.

**Table 1:** Primers used in fluorescence quantitative PCR.

Name	Primer pair
PTEN	F: 5′CAGAGCGAGGGCATCAC-3′
	R: 5′GCAGGAAATCCCATAGCAATAA-3′
Akt	F: 5′GTGCTGGAGGACAATGACTA-3′
	R: 5′AGCAGCCCTGAAAGCAAGGA-3′
PI3K	F: 5′ATGGGGATGATTTACGGC-3′
	R: 5′TCTCCTTTGTTCTTGTCTTTGA-5′
DJ-1	F: 5′ACTGCGTTCGGAATTGCTGCAT-3′
	R: 5′AGTCCAGTTGACCGTTGACCTTAACCAA-5′
*β*-Actin	F: 5′CTTCCTTCCTGGGCATG-3′
	R: 5′GTCTTTGCGGATGTCCAC-3′

**Table 2:** Effects of curcumol treatment on percentage of apoptotic human hepatocellular carcinoma HepG2 cells.

Time	Concentration (*μ*g/mL)	Percentage of early apoptotic cells (%)	Percentage of late apoptotic cells (%)
24 h			
	10	1.54 ± 0.52	1.31 ± 0.33
	30	2.06 ± 0.58	2.75 ± 0.49
	100	4.39 ± 0.67^#^	6.14 ± 1.76^#^
	DMSO group	0.83 ± 0.43^∗^	0.42 ± 0.19^∗^

48 h			
	10	3.14 ± 0.54	2.55 ± 0.46
	30	4.07 ± 0.75	4.36 ± 0.59
	100	6.27 ± 1.38^#^	8.18 ± 0.87^#^
	DMSO group	0.96 ± 0.37^∗^	0.57 ± 0.36^∗^

72 h			
	10	4.35 ± 0.63	5.24 ± 0.86
	30	6.27 ± 1.32	6.46 ± 1.11
	100	9.27 ± 1.64^#^	11.35 ± 2.09^#^
	DMSO group	1.04 ± 0.47^∗^	1.29 ± 0.47^∗^

^∗^ *p* < 0.05 vs. the DMSO group at the same time point, with a significant difference, and ^#^*p* < 0.05 vs. the 10 *μ*g/mL group at the same time point, with a significant difference.

**Table 3:** Inhibition of curcumol in varying concentrations and different treatment times on the growth of human hepatocellular carcinoma HepG2 cells.

Concentration (*μ*g/mL)	Growth inhibition rate (%)		
	24 h	48 h	72 h
10	5.25 ± 0.64	9.26 ± 1.37	13.35 ± 2.14
30	8.32 ± 1.35	14.06 ± 2.54	19.69 ± 2.74
100	12.36 ± 2.35	21.86 ± 2.97	31.45 ± 3.97

Note. (1) There are significant differences among different groups at the same time point (*p* < 0.05). (2) There are significant differences at different time points in the group treated with the same concentration (*p* < 0.05).

**Table 4:** Effects of curcumol in varying concentrations and different treatment times on protein expressions in human hepatocellular carcinoma HepG2 cells.

Time	Concentration (*μ*g/mL)	PTEN	p-Akt	DJ-1	PI3K
24 h					
	10	0.29 ± 0.08	0.45 ± 0.21	0.34 ± 0.13	0.51 ± 0.17
	30	0.35 ± 0.18	0.31 ± 0.13	0.25 ± 0.11	0.49 ± 0.23
	100	0.56 ± 0.21^#^	0.14 ± 0.06^#^	0.13 ± 0.06^#^	0.26 ± 0.15^#^
	DMSO group	0.15 ± 0.07^∗^	0.52 ± 0.18^∗^	0.43 ± 0.15^∗^	0.59 ± 0.28^∗^

48 h					
	10	0.37 ± 0.14	0.38 ± 0.21	0.31 ± 0.14	0.42 ± 0.14
	30	0.42 ± 0.16	0.27 ± 0.11	0.18 ± 0.12	0.36 ± 0.17
	100	0.65 ± 0.19^#^	0.13 ± 0.07^#^	0.09 ± 0.05^#^	0.21 ± 0.11^#^
	DMSO group	0.13 ± 0.09^∗^	0.87 ± 0.32^∗^	0.53 ± 0.14^∗^	0.67 ± 0.23^∗^

72 h					
	10	0.48 ± 0.14	0.32 ± 0.11	0.23 ± 0.17	0.28 ± 0.13
	30	0.56 ± 0.22	0.15 ± 0.12	0.14 ± 0.06	0.17 ± 0.09
	100	0.87 ± 0.31^#^	0.10 ± 0.09^#^	0.10 ± 0.07^#^	0.09 ± 0.04^#^
	DMSO group	0.13 ± 0.07^∗^	0.74 ± 0.23^∗^	0.54 ± 0.26^∗^	0.53 ± 0.24^∗^

Note: ^∗^comparison with the control group, with a significant difference at the same time point (*p* < 0.05); ^#^comparison between the 100 *μ*g/mL group and the 30 *μ*g/mL group or the 10 *μ*g/mL group, with a significant difference (*p* < 0.05).

**Table 5:** Effects of curcumol in different concentrations and different treatment times on gene expressions in human hepatocellular carcinoma HepG2 cells.

Time	Concentration (*μ*g/mL)	PTEN	Akt	DJ-1	PI3K
24 h					
	10	0.37 ± 0.11	0.48 ± 0.20	0.45 ± 0.12	0.43 ± 0.21
	30	0.42 ± 0.16	0.35 ± 0.16	0.36 ± 0.12	0.36 ± 0.15
	100	0.59 ± 0.24^#^	0.39 ± 0.07	0.19 ± 0.07^#^	0.24 ± 0.11^#^
	DMSO group	0.17 ± 0.09^∗^	0.59 ± 0.15	0.47 ± 0.13^∗^	0.64 ± 0.23^∗^

48 h					
	10	0.44 ± 0.18	0.36 ± 0.22	0.30 ± 0.12	0.40 ± 0.19
	30	0.53 ± 0.24	0.34 ± 0.12	0.19 ± 0.14	0.30 ± 0.12
	100	0.69 ± 0.21^#^	0.45 ± 0.07	0.08 ± 0.06^#^	0.15 ± 0.08^#^
	DMSO group	0.15 ± 0.08^∗^	0.56 ± 0.25	0.55 ± 0.21^∗^	0.67 ± 0.23^∗^

72 h					
	10	0.53 ± 0.24	0.47 ± 0.10	0.24 ± 0.13	0.26 ± 0.09
	30	0.62 ± 0.25	0.48 ± 0.13	0.12 ± 0.04	0.14 ± 0.05
	100	0.79 ± 0.28^#^	0.59 ± 0.03	0.08 ± 0.03^#^	0.06 ± 0.02^#^
	DMSO group	0.19 ± 0.06^∗^	0.61 ± 0.24	0.52 ± 0.22^∗^	0.59 ± 0.31^∗^

Note: ^∗^comparison with the control group, with a significant difference at the same time point (*p* < 0.05); ^#^comparison between the 100 *μ*g/mL group and the 30 *μ*g/mL group or the 10 *μ*g/mL group, with a significant difference (*p* < 0.05).

## Data Availability

The datasets used and/or analyzed during the current study are available from the corresponding author on reasonable request.
